# Improvement of Speech Recognition Technology in Piano Music Scene Based on Deep Learning of Internet of Things

This article has been retracted.

**DOI:** 10.1155/2022/4024511

**Published:** 2022-07-13

**Authors:** Jie Bai

**Affiliations:** Department of Music, Xi'an Shiyou University, Xi'an 710065, Shaanxi, China

## Abstract

The main goal of speech recognition technology is to use computers to convert human analog speech signals into computer-generated signals, such as behavior patterns or binary codes. Different from speaker identification and speaker confirmation, the latter attempts to identify or confirm the speaker who uttered the speech rather than the lexical content contained in it. The short-term idea is that it should be able to record the musical sound played by the user with a certain musical instrument, then extract the note and duration information from it, and finally generate the corresponding MID file according to the MIDI standard, which can set the type of musical instrument in advance to complete the function of musical sound transformation, such as playing with a harmonica, and playing the MID at the end is the piano sound. With the rapid development of the mobile Internet, fields such as machine learning, electronic communication, and navigation have placed high demands on real-time and standard text recognition technology. This paper merges the sound of visual music into text-based data set training, uses the exported scanner features for model training, uses the model to extract features, then uses the features for prior training, and then uses pretraining. DNN results show that the combined training of target prevention and expansion plans, by replacing long-term and short-term memory networks, end-to-end speech recognition programs, and behavioral tests organized by mobile devices, can provide a larger receptive field combined with expanded convolution instead of long and short periods. The experimental results show that when the input sampling point is 2400, it can be seen that the convergence speed of the model becomes slower with more than 90 iterations and the loss of the model on the verification set increases with the increase in the number of iterations. This shows that the model in this paper can fully meet the needs of speech recognition in piano music scenes.

## 1. Introduction

There have been many advances in speech recognition technology, such as the fact that people can talk to Siri on their iPhones. There has also been progress in another technology-related field, music tracking and recognition. For example, WeChat can shake one-shake to search for songs, and the mobile phone can quickly find the song name according to the “listened” music and display the lyrics synchronously, indicating that the music sound recognition technology is also becoming more and more into people's lives. Technology is indeed changing people's lives all the time. The Internet of Things realizes the ubiquitous connection between things and things and things and people and realizes the intelligent perception, identification, and management of objects and processes [1]. Music recognition technology is the hub connecting musical instruments and real music. Through music recognition technology, the computer can automatically recognize the melody, noise, genre, theme, and other information of the song.

Technological development not only meets existing needs but also creates demand because technological development has found the possibility of solving some problems that were previously unimaginable. As a piano lover, the author wants to play her favorite tunes through the piano, which can be recorded, edited, processed, recreated, and then shared or entertained. Traditional and nontraditional network models have achieved excellent results in text recognition research, but they have encountered bottlenecks. Like standard neural network upgrade algorithms, traditional network modeling methods are not suitable for simple-scale networks. The starting point of the BP algorithm is randomly selected [2]. The depth of the network will make the learning of parameters fall into a local optimum. The advent of deep learning reduces the possibility of falling into a better environment and can improve the capabilities of the model [3]. Deep learning can be seen as an extension of machine learning, and it is also the development trend of traditional networks. Deep learning is a multilayer perceptron with many hidden levels. By combining the characteristics of the underlying data with a standard data distribution system, the high characteristics expression of the data can be determined. In addition, this research provides a reference for speech recognition technology in special scenarios.

For speech recognition methods in different environments, experts at home and abroad have conducted many studies. Gordon-Salant and Cole aim to determine whether the working memory has different breadths and whether it performs differently in noisy speech recognition tests [4]. Hizlisoy et al. proposed CLDNN [5]. Vo Q N et al. proposed the detection of curved staff based on RANSAC, divided the staff into sub-regions for correction by biquadratic transformation, and used run-length coding to identify musical [6]. Sotoodeh et al. believe that music symbol recognition provides high accuracy in identifying symbols [7]. In order to evoke reaction emotions, Bo et al. designed a three-stage experimental paradigm of long-term musical stimulation through time analysis and inspiration-maintenance decline [8]. Chin et al. proposed a new music emotion content recognition system, which integrates three computational intelligence tools, namely, the hyper-rectangular composite neural network (HRCNN), fuzzy system, and PSO. They extracted original features from each piece of music and cleared rules are transformed into fuzzy rules with confidence factors [9]. The spectrum markers is intended to achieve robustness, so Gutiérrez and Garcia define and established an appropriate fitness evaluation method by converting its highly correlated parameters into various genes [10]. However, due to the lack of relevant voice data in these studies, there are also some controversies in the methods used, resulting in the related results not being recognized by the public. The conclusions of these studies have not been fully explained, so this part of the content is still open to question.

Research on the Internet of Things has been going on, and Zhoa et al. outlined a set of requirements for IoT middleware and conducted a comprehensive review of existing middleware solutions against these requirements [11]. Bisharad and Laskar surveyed over a hundred IoT smart solutions on the market and carefully studied them to determine the technologies, functions, and applications used [12].

Compared with the traditional training model, the deep training model has great advantages and can overcome the limitations of the shallow model's limited computing power and general capacity limitations. However, the deep model also faces some difficulties. The amount of data to be learned during training is very large, but the noise of the training data will be affected during the training process, and the noise performance will be revealed. In order to solve this problem, this paper proposes two methods to improve the optimization process after training, namely, random exit method and random feature connection, to reduce the potential training data adopted by the deep model. As the training data are reduced, the compatibility with the depth model is reduced, and the weight update process is more independent; instead of relying on the function of the hidden segment of the fixed focus, the training effect is improved. This paper fuses the sound of visual music into a text-based dataset training, uses the exported scanner features for model training, uses the model to extract features, then uses these features for pretraining, and then uses pretraining.

## 2. Research Methods of Speech Recognition Technology in Music Scenes

### 2.1. Speech Recognition

The piano scene is a special kind of scene, and how to perform speech recognition in this scene is a more difficult problem. Voice recognition technology can detect human-computer interaction. With the development of high and new technology, the competition in the application of speech recognition technology is becoming more and more fierce and it has high technical and development capabilities in many application fields and application expectations. Deep learning is a new research in machine learning research that can simplify the process of interpreting human brain data [13, 14]. In-depth phonetic research has become a field of recognition research, and the research field is expanding [15]. Voice recognition generally has two working modes: recognition mode and command mode. The realization of the voice recognition program will also adopt different types of programs according to the two modes.

Audio data are a part of continuous audio signals. If you observe them for a long time, you will see these signals constantly changing between different states. If you observe them for a short time, you can regard them as a stable state [13]. The speech recognition system is mainly composed of four modules: audio feature output, audio model, language model, and decoder. The audio feature output unit processes the predefined speech signal, first changes the input signal from the time zone to the frequency band, and then uses an appropriate method to remove the best possible feature of the audio model [16, 17]. The audio model must input the feature vector mentioned above to calculate the matching of the speech signal and the phoneme. The language model records the probability of a word by reading a large number of words and calculates the probability that each word corresponds to a phoneme. The decoder unit combines the model acoustics, model language, and vocabulary information to calculate the sequence most likely to match the vector attribute input [18].

The format wave data obtained by the audio signal sampling and comparison are sent to the preaudio output unit, and structured balls of various sizes are output for later audio model training [19, 20]. Good audio features not only retain information related to speech and content exposure and eliminate speaker factors, area, and noise interference but also use the smallest possible parameter size without losing detailed information, which is very useful to achieve better training results [21]. Audio sampling rate refers to how much the recording device samples the analog signal per unit time. The higher the sampling frequency, the more realistic and natural the waveform of the mechanical wave will be. The outline of the sound event recognition system is shown in Figure 1.

Traditional speech recognition systems are usually divided into several parts, such as extracting and learning audio features, audio sampling, and language modeling [14]. Each module is optimized separately, resulting in a tight connection of input and output, detecting more errors, and wasting more application resources. Studies have shown that learning features play an important role in speech recognition systems [10, 22]. The deep network combines feature learning and process optimization, thereby reducing the number of modules in the word recognition system. A text recognition system that uses algorithms to complete everything from text input to word processing is called an end-to-end text recognition system. Although the current end-to-end word recognition system does not surpass the traditional word recognition process in practice, it has attracted more and more researchers [23].

The data sharing module is the first and most important part of designing an event recognition system [24, 25]. To measure effectiveness and create a class, the initial database is usually divided into a training program, a verification program, and a set of tests. Among them, the training plan and certification plan are necessary, and the existence of the test plan depends on the specific situation [26]. As the name implies, the training plan is used to train the trainees. Since the programmer's work is always consistent with the size of the training plan, most of the data in the initial database will be split into the training plan. Using the verification system in the training process of the classifier can observe the operation of the classifier in real time during the training process, thereby effectively adjusting the lifespan or characteristics of the classifier. In addition to the certification system, the test system is used after programmer training. The index obtained by the classifier in the test system can indicate the final performance of the classifier [27].

### 2.2. Voice Enhancement Technology

The current speech recognition technology has the highest detection rate when the external noise level is low, and the normal detection rate of the recognition system will drop rapidly when the external noise level is high. In order to maximize the ability of the text recognition system in a viscous noise environment, the screen correction unit on the front end of the speech recognition system applies a variety of text enhancement algorithms, such as training jointly with the original samples by standard methods or advanced training methods and also based on confusion (mixup) interpolation text and labels for enhancement [28]. The speech recognition system mainly has five components, and the training phase mainly includes training an acoustic model and a language model. The principle of the speech recognition system is shown in Figure 2.

Due to the evolution, the high-frequency side of the received audio signal will drop by 6 dB per octave after it is generated, while the noise signal is the opposite. This makes the low-noise signal of the speech signal larger and the low-frequency signal reaching the speaker is smaller, which makes the transmission difficult [29]. In order to solve this problem, advanced technology will be used in the early stage of the audio signal to increase the high-frequency component of the audio signal to compensate for the loss. The voice waveform before and after preemphasis is shown in Figure 3.

The preprocessing module is to prepare for the next feature export part. It mainly includes the following functions: first, the input data are modified in the comprehensive standardized storage system by means of review, bit size adjustment, and size measurement to ensure data consistency. For example, raw data will definitely be combined with stereo and mono audio. Second, there will be a certain amount of noise in the original data, and noise always interferes with the operation of the classifier, so corresponding noise reduction must be increased. Third, for the purpose of data processing, the object data already exist and the audio data will be preemphasized, windowed, and framed. In addition, signal systems such as endpoint detection and time series are also important links in the previous section.

The feature extraction module includes the core of the entire event recognition system [30]. “Data and structure define the upper limit of machine learning, and models and algorithms can only be as close as possible to this upper limit.” The feature extraction here refers to the data received through attribute derivation. The speech recognition problem is mainly a machine learning problem, so the feature derivation module is very important. Images are information that can effectively show the nature of the data and help predict the results. Product removal refers to the process of converting raw data into training data for a good model. Sometimes, even a simple model can achieve good results. In audio event recognition, the most common features including fundamental frequency, uniformity, optical center, short-term power, group power side, zero speed, short-range, Mel cepstrum detector, LPC line predictor, LPC and LPCst systems, and LSP line parameters are equal.

### 2.3. Deep Learning

We adjusted the two-dimensional convolutional network that performed well in images to a one-dimensional convolutional network that is more suitable for speech signals and used the one-dimensional convolutional neural network model and the long-short-term memory network model to implement speech acoustic feature extraction, speech separation, and voice recognition. Convolutional neural network is a kind of feedforward neural network with deep structure including convolution calculation and is one of the representative algorithms of deep learning. The convolutional neural network further cancels the full connection between the hidden layers of the feedforward neural network and replaces it with a partial connection with a weight distribution. Convolution is an important line in mathematical calculations. Valid convolution, same convolution, and full convolution are three commonly used convolution operations in digital signal processing.

#### 2.3.1. Valid Convolution

(1) $$\begin{array}{c} \left\{\begin{array}{c} y=\text{conv}\left(x,w,\text{valid}\right)=\left(y\left(1\right),...,y\left(n-m+1\right)\right),\\ y\left(t\right)=\sum_{i=1}^{m}x\left(t+i-1\right)w\left(i\right), \end{array}\right. \end{array}$$

where *t*=1,2,…, *n* − *m*+1 and *t*=1,2,…, *n* − *m*+1.

#### 2.3.2. Full Convolution

(2) $$\begin{array}{c} \left\{\begin{array}{c} y=\text{conv}\left(x,w,\text{full}\right)=\left(y\left(1\right),...,y\left(n-m+1\right)\right),\\ y\left(t\right)=\sum_{i=1}^{m}x\left(t-i+1\right)w\left(i\right). \end{array}\right. \end{array}$$

#### 2.3.3. Same Convolution

(3) $$\begin{array}{c} y=\text{conv}\left(x,w,\text{same}\right)=\text{center}\left(\text{conv}\left(x,w,\text{full}\right),n\right). \end{array}$$

The returned structure is the central part of the full convolution with the same size as the input signal *x*, as shown in Figure 4.

According to the valid convolution, the size of the output signal obtained by combining the step size and the filling operation is

(4) $$\begin{array}{c} \left\{\begin{array}{c} y=x*w\in S^{u\times v},\\ u=\left[\frac{n-s+2*\text{Zeropadding}}{\text{Stride}}\right],\\ v=\left[\frac{m-k+2*\text{Zeropadding}}{\text{Stride}}\right]. \end{array}\right. \end{array}$$

Pooling refers to a down-sampling operation; that is, in a small area, a specific value is taken as the output value of the area, so the pooling layer is also called a down-sampling layer. Maximum pooling and mean pooling can be expressed as

(5) $$\begin{array}{c} a_{ij}=\max\left(x_{i+l,j+l},x_{i+l+1,j+l},...,x_{i+l+n-1},x_{j+l+n-1}\right),\\ a_{ij}=\frac{1}{n*n}\sum_{a=i+l,b=j+l}^{n-1}x_{ab}, \end{array}$$

where *a*_*ij*_ is the output value of the neuron after passing through the pooling layer, *n* is the pooling radius, and *l* is the step length of the pooling.

Convolution is a linear function. In the calculation process, addition, and multiplication are only included in the model adjustment process. The vector in the linear integer space must be mapped to the linear part of the space through nonlinear conversion. The activation function is the method to introduce nonlinearity. The current common activation function types are shown in Figure 5.

The hard limit function (hardlim) and its expression is as follows:

(6) $$\begin{array}{c} y=f\left(x\right)=\left\{\begin{array}{c} \begin{array}{cc} 0, & x<0, \end{array}\\ \begin{array}{cc} 1, & x\geq 0, \end{array} \end{array}\right. \end{array}$$

Or

(7) $$\begin{array}{c} y=f\left(x\right)=\text{sgn}\left(x\right)=\left\{\begin{array}{cc} -1, & x>0,\\ 1, & x\geq 0, \end{array}\right. \end{array}$$

Among them, sgn(·) is called a symbolic function, formula (6) is a single limit function, and formula (7) is a double limit function.

The Sigmoid function was widely used in neural networks before, and its expression is as follows:

(8) $$\begin{array}{c} y=f\left(x\right)=\frac{1}{1+e^{-\lambda x}}. \end{array}$$

The Gaussian radial basis function and its expression is shown in the following formula:

(9) $$\begin{array}{c} y=f\left(x\right)=\exp\left(-\frac{x^{2}}{\delta^{2}}\right). \end{array}$$

Rectified linear units (ReLUs) are expressed as

(10) $$\begin{array}{c} y=f\left(x\right)=\max\left(0,x\right). \end{array}$$

The most commonly used function in neural networks is the sigmoid function. The derivation of the sigmoid function is very simple, but when the independent variable is far away from the origin of the coordinate, the slope of the function decreases rapidly and tends to 0, resulting in “gradient disappearance.”

The core design of the network mainly includes three gates, namely, input gate, forget gate, and output gate.

Input gate: the main purpose of this gate is to determine how much information in the input tX remains in *C*_*t*_ , and the realization formula is

(11) $$\begin{array}{c} \left\{\begin{array}{c} i_{t}=\sigma \left(Wi*\left[h_{t-1},xt\right]+b_{i}\right),\\ C=\tanh\left(W_{C}*\left[h_{t-1},xt\right]+b_{C}\right), \end{array}\right. \end{array}$$

where *i*_*t*_ is the input of the input gate at time *t*, through the input gate, the corresponding *C*_*t*_ times in the input are retained, *W* represents the weight matrix, and *b* represents the bias.

### 2.4. Evaluation Methods and Indicators

In machine learning and model recognition problems, modeling the performance of a model or algorithm requires a certain degree of accuracy and efficiency. Similarly, when calculating an event recognition system, especially when comparing different algorithms and different features, some clues that can accurately indicate your performance can not only help a person understand and identify the pros and cons of these algorithms (or features), in order to further improve .

The most common evaluation criteria for classification models are accuracy and error rate. As the name implies, the error rate is the part of the number of samples that is not divisible by the total number of samples, and the normal rate is the part of the total number of samples that are correct. For data set *D*, the error rate is defined as follows:

(12) $$\begin{array}{c} E\left(f;D\right)=\frac{1}{M}\sum_{n=1}^{M}P\left(f\left(x_{n}\right)\neq y_{n}\right). \end{array}$$

Among them, *M* is the total number of samples in the data set *D*, *x*_*n*_ is the feature of the nth sample, and *y*_*n*_ is the label.

The accuracy is defined as

(13) $$\begin{array}{c} Ac\left(f;D\right)=\frac{1}{M}\sum_{n=1}^{M}P\left(f\left(x\right)=y_{n}\right)=1-E\left(f;D\right). \end{array}$$

Accuracy and error rates can usually better reflect the performance of a classification model. The higher the accuracy and the lower the error rate, the better the performance of the model.

Error backpropagation is a supervised learning method, we express it as follows:

(14) $$\begin{array}{c} e\left(n\right)=d\left(n\right)-y\left(n\right)=\sum_{j\in C}d_{j}\left(n\right)-y_{j}\left(n\right), \end{array}$$

where *d*_*j*_(*n*) is the *j*th component of *d*(*n*). Then, the cost function can be expressed as follows:

(15) $$\begin{array}{c} \varepsilon \left(n\right)=\sum_{j\in C}\varepsilon_{j}\left(n\right)=\frac{1}{2}\sum \varepsilon_{j}^{2}\left(n\right). \end{array}$$

The cost function *ε*(*n*) is used as the learning evaluation of neural network learning, and the weight of each neuron in the network can be used to reduce the cost function to achieve the effect of training the network. Assuming that Δ*w*_*ij*_ is the adjustment change of weight *w*_*ij*_ in each weight adjustment process, then the update of weight *w*_*ij*_ is calculated as follows:

(16) $$\begin{array}{c} w_{ij}=w_{ij}+\Delta w_{ij}. \end{array}$$

Since *w*_*ij*_ is proportional to the partial derivative and *λ* is the learning rate, then Δ*w*_*ij*_ can be calculated as follows:

(17) $$\begin{array}{c} \Delta w_{ij}=-\lambda \frac{\partial \varepsilon \left(n\right)}{\partial w_{ij}}. \end{array}$$

After that, using the chain derivation rule, the formula can be expanded as

(18) ∂εn∂wij=−ejn·fvjn·yni.

After the local gradient *δ*_*j*_ is calculated, the weights in the network can be updated and calculated:

(19) $$\begin{array}{c} \frac{\partial \varepsilon \left(n\right)}{\partial y_{j}\left(n\right)}=-\sum_{k}e_{k}\left(n\right)\cdot f\left(v_{k}\left(n\right)\right)\cdot w_{ij}=-\sum_{k}\delta_{k}w_{ij}. \end{array}$$

At this point, by completing the solution of the local gradient, the amount of change in the network weight is obtained, so as to achieve the purpose of adjusting the network weight, so that the network can continue to be trained.

## 3. Speech Recognition Experiment and Analysis

### 3.1. Experimental Setup

The audio samples are divided into frames, each frame is 0.02 seconds long, and the frame overlap rate is 50%. After that, the features are extracted in units of frames, and after the feature extraction is completed, the overall data set is normalized. The hyperparameters of the network under different data sets are shown in Table 1.

In order to better analyze the performance of the model, 4 different classifiers are introduced and compared. The recognition rate of the model is compared with the ratio as shown in Table 2.

It can be seen that both belong to deep learning models, but KNN is a cyclic neural network with a special system. It is very good at processing time series data and can efficiently extract features from individual data to achieve excellent operation recognition. .

Figure 6 is the confusion matrix of the KNN model on the ESC-10 data set, which comprehensively shows the classification of the KNN model in each category. Among them, DB, RA, SW, BC, CT, PS, HP, CS, RT, and FC represent dog barking, rain, ocean waves, baby crying, hour hand turning, human sneezing, and helicopter turning, respectively. The sound of chainsaws was flames and music. KNN is the neighbor algorithm, or the *K* nearest neighbor classification algorithm, which is one of the simplest methods in data mining classification technology.

The advantage of KNN network is that it can solve long-term reliability problems with fewer parameters, avoid tilt loss and sudden explosion problems, and can effectively extract data from individual data. Therefore, compared to models such as SVM and DNN, the KNN network has achieved better recognition in both ESC and TUT data systems.

We analyzed the effect of signal decomposition and calculated the sparsity required to obtain different DeSNRs, as shown in Table 3.

It can be seen from the table that the gain-to-noise ratio of the signal-to-noise ratio is 8.1, but after nearly 80,000 iterations, the entire iteration process takes 110 seconds, which consumes a lot of time and memory.

It should be pointed out that these feature types do not appear separately. It is very likely that multiple changes will occur in one music version at the same time. The above version types and music features can be combined, as shown in Table 4. This brings more challenges to music version identification.

### 3.2. Recognition Effect in Music Scene

In the test, the text part of the text sample needs to be extracted first, and the method used is to remove the characteristic parameters of the Mel cepstrum coefficient and MMFC coefficient of the text sample. The basic principle of MMFC parameter export is: first obtain a continuous speech, perform preemphasis, framing and windowing operations on the function in the template, and then Fourier transform (FFT), use Mel filter to smooth the spectrum, and then logarithm Operate and separate the cosine transform to obtain the MFCC parameters.

Before speech feature extraction, the speech signal is sampled first, and the time domain graph of the original speech signal and the frequency spectrum of the original speech signal are drawn. Taking a music scene as an example, Figures 7(a) and 7(b) are the time domain diagram of the original voice signal and the frequency spectrum diagram of the original voice signal, respectively.

It can be seen that in the selected scene, because it is in the field of music, the system recognition error rate is too high for continuous noise levels and noises that are highly confused with text. Therefore, we use the Internet of Things deep learning technology to improve and learn related languages. Reduce the influence of noise in the music scene. When sampling positions of different frame lengths are used in input, in order to ensure the performance of the model in the training system and the verification was program. We collected 4 types of frame length speech recognition situations.

The orange curve is used to represent the model work in the verification system, and the blue side is used to represent the model work in the training system. The number on the left represents the change during the training process. The correct shape represents the variation of the standard model in the number of iterations, the horizontal position of the iteration number, and the vertical position with the correct rate. We first perform statistics on 560 sampling points, as shown in Figure 8.

We performed statistics on 1600 sampling points, and the results are shown in Figure 9.

We performed statistics on 2400 sampling points, and the results are shown in Figure 10.

It can be seen from Figures 9 and 10 that the model has gone through more iterations, has jumped out of the local optimal solution, and optimized the network parameters in the direction of less loss. When the input sampling point is 2400, it can be seen that the convergence speed of the model slows down, and the iteration exceeds 90 times. The loss of the model on the verification set increases with the increase in the number of iterations, which leads to the overfitting of the model.

## 4. Discussion

Optical music recognition (OMR) can be divided into three main stages, line detection and removal, music symbol recognition, and music symbol detection and segmentation. The specificity of this method is 99.71%, which is the existing method. In addition, recall and f-measure are only slightly smaller than the best methods in terms of accuracy.

As an integral part of the audio system, speech recognition technology uses audio signals to understand the environment and judge many complex situations in the area. Compared with video and video signals, audio signals are not restricted by conditions such as angle, light, and ground, and require very little storage space and computers. They are ideal for human-to-human interaction computers and are therefore most suitable for security. It has a wide range of application expectations in human-computer interaction and other fields.

A key issue is an in-depth study on how to obtain a large amount of point data. Research shows that the larger the data set applied to the deep learning network, the better the impact. However, it is not easy to obtain a large amount of labeled data. Therefore, in practical applications, it is necessary to study how to use a limited amount of data to achieve the best possible filtering effect.

When deep learning is trained in a small sample database, it is prone to insufficient training and unsatisfactory training effects. Focusing on deep learning problems is more likely to occur when training a small amount of data. We propose a new level of deep learning improved method to make the weight update more independent, have the hidden segment of the stable neurons, and reduce the dependence between neurons, to obtain a more stable density and increase the depth of learning. Backpropagation algorithm and deep belief network construct network models, respectively, construct and test network models. BP neural network and deep belief network are used to verify the verbal identity of a single word, and then two methods of refinement and optimization are introduced into the deep belief network and compared. Tests show that the speech recognition rate of deep learning is higher than that of traditional networks.

Deep networks have achieved great success in word recognition, partly because of the flexibility of the DNN model in learning complex signal processing techniques. However, this flexibility will cause significant distortion, which will cause the performance of the speech recognition system to drop sharply under the influence of high noise. In this article, we start with the research of high-noise speech training, explore how to inject noise and noise training, and propose a new noise training method to improve the ability of the speech recognition system to recognize DNN problems.

## 5. Conclusion

A complete music recognition not only includes direct information such as rhythm, dynamics, notes, and duration but also indirect information such as instrument type, chord name, and music style. An ideal music sound recognition system can record the live music tones as musical scores and save them. And output sheet music, which can be used to assist composition, music education, song search, life entertainment, and so on. The robustness of the speech recognition system is the primary issue that restricts the operation of the speech recognition system. This paper first studies the speech processing algorithm used to generate the front-end signal and proposes the optimization of the Bayesian proposition based on the concept of obtaining density under the Chi distribution. Start with high-noise speech training, discuss how to induce noise and noise training, and design a new noise training method to enhance the speech recognition cognitive ability of DNN training effects. Perform previous DBN training on the exported parts. After the previous training is completed, the randomly generated production levels are integrated, and the backbone algorithm is used to distinguish all the weights in the network in detail. Therefore, using the DBN model created by previous training in the DNN training process will give the DNN the best starting weight, and then the best model can be trained. Of course, the research in this article also has some shortcomings. Traditional speech enhancement algorithms usually require some assumptions. However, in some environments, these assumptions may not be fully satisfied, so it will lead to a certain degree of degradation in the performance of the enhanced algorithm. Due to the wide range of research in the field of speech recognition, the needs of practical applications are also an important basis for guiding future research work.

## Figures and Tables

**Figure 1:** Overview of the sound event recognition system.

**Figure 2:** Principle of the speech recognition system.

**Figure 3:** Waveform (a) before and (b) after preprocessing.

**Figure 4:** Convolution process. (a) One-dimensional convolutional diagram; (b) convolution process.

**Figure 5:** Common activation functions: (a) hard limit function; (b) sigmoid function; (c) hyperbolic tangent function.

**Figure 6:** Confusion matrix on the KNN dataset.

**Figure 7:** Time domain and frequency spectrum of speech signal.

**Figure 8:** 560-sampling point performance impact.

**Figure 9:** 1600-sampling point effect.

**Figure 10:** 2400-sampling point changes.

**Table 1:** Hyperparameters under different data sets.

Hyperparameters	Dataset		
	ESC-10	ESC-50	TUT
Dropout ratio	0.18	0.25	0.47
Learning policy	Fixed	Fixed	Stepwise
Momentum	0.025	0.005	0.002
Weight decay	0.89	0.94	0.88
Learning rate	Adam	SGD	SGD
Mini-batch	0.05	0.01	0.02
Optimizer type	31	117	31
Epochs	49	78	149

**Table 2:** Recognition rate of different classifiers.

Classifier	Dataset		
	ESC-10 (%)	ESC-50 (%)	TUT (%)
GMM	61.8	36.3	77.7
SVM	66.4	38.5	82.1
DNN	69.1	41.8	83.5
KNN	67.9	39.5	81.8

**Table 3:** Sparsity required for different DeSNRs.

DeSNR	0.4	1.3	1.8	2.1	2.6	3.1	4.1	4.7	5.2	6.2	7.4
Sparsity	10	100	200	300	500	900	2800	5800	8800	19K	40 K
Decomposition time/s	0.15	0.17	0.24	0.29	0.79	1.68	4.82	9.51	13.2	30.4	61.7

**Table 4:** The relationship between music element changes and version types.

Type label	Timbre	Speed	Beat	Structure	Tune	Chord	Lyrics	Noise
Ripping	Y							Y
Instrumental music	Y						Y	Y
Mash up	Y						Y	Y
On-site	Y			Y				Y
Vocal	Y	Y	Y					Y
Mock up	Y	Y	Y		Y	Y	Y	Y
Standard song	Y	Y	Y	Y	Y	Y		Y
Skewers	Y	Y	Y	Y	Y	Y		Y
Mix	Y	Y	Y	Y	Y	Y	Y	Y
Quote	Y	Y	Y	Y	Y	Y	Y	Y

Y indicates that there may be changes in the musical element.

## Data Availability

No data were used to support this study.
